# MiR-30a-5p Antisense Oligonucleotide Suppresses Glioma Cell Growth by Targeting SEPT7

This article has been retracted.

**DOI:** 10.1371/journal.pone.0055008

**Published:** 2013-01-28

**Authors:** Zhifan Jia, Kun Wang, Guangxiu Wang, Anling Zhang, Peiyu Pu

**Affiliations:** 1 Department of Neurosurgery, Tianjin Medical University, General Hospital, Tianjin Neurolgical Institute, Laboratory of Neuro-Oncology, Key Laboratory of Post-Trauma Neuro-Repair and Regeneration in Central Nervous System, Ministry of Education, Tianjin Key Laboratory of Injuries, Variations and Regeneration of Nervous System, Tianjin, People’s Republic of China; 2 Department of Neurosurgery, Hangzhou Xiasha Hospital, Sir Run Run Shaw Hospital, Medical College, Zhejiang University, Hangzhou, People’s Republic of China; City of Hope National Medical Center and Beckman Research Institute, United States of America

## Abstract

MicroRNAs (miRNAs) are small noncoding RNAs that regulate gene expression by targeting the mRNAs of hundreds of human genes. Variations in miRNA expression levels were shown to be associated with glioma. We have previously found miR-30a-5p overexpression in glioma cell lines and specimens. Bioinformatics analyses predict that several miRNAs, including miR-30a-5p, are involved in the post-transcriptional regulation of SEPT7. SEPT7 is a member of the septin family, which is a highly conserved subfamily of GTPases implicated in exocytosis, apoptosis, synaptogenesis, neurodegeneration and tumorigenesis. Our previous study has also demonstrated that SEPT7 expression is decreased in astrocytic gliomas with different grades and plays a tumor suppressor role. In the present study, we knocked down miR-30a-5p with antisense oligonucleotide (miR-30a-5p AS) in LN229 and SNB19 glioblastoma(GBM) cells, and found that cell growth and invasion were inhibited, while apoptosis was induced. miR-30a-5p AS treated cells showed upregulation of SEPT7 and downregulation of PCNA, cyclin D1, Bcl2, MMP2 and MMP9. In contrast, when miR-30a-5p mimics were transfected into LN229 and SNB19 GBM cells, cell growth and invasion were promoted and the expression of relevant proteins increased. Meanwhile, the effect of miR-30a-5p mimics on glioma cells can be reversed by transfection of SEPT7 construct. Additionaly, miR-30a-5p directly targeting SEPT7 was identified by the reporter gene assay. Our study demonstrates,for the first time, that miR-30a-5p is a bona fide negative regulator of SEPT7 and the oncogenic activity of miR-30a-5p in human gliomas is at least in part through the repression of SEPT7.

## Introduction

Malignant gliomas, such as glioblastoma multiforme (GBM), are the most common and aggressive malignant primary brain tumors. Despite the advances in surgery, radiation therapy, and chemotherapy, the prognosis of patients with GBM has not been improved significantly over the past 20 years [1]. It is imperative to have a detailed and comprehensive understanding of the molecular pathogenesis of the gliomas for developing novel strategies in treatment.

miRNAs are small, evolutionarilly conserved noncoding RNA molecules, Recent studies have shown that the expression of many miRNAs are deregulated in a variety of cancers, including lymphoma, colorectal cancer, lung cancer, breast cancer, papillary thyroid carcinoma, hepatocellular carcinoma and glioblastoma [2]–[8]. Regarding the role of miRNAs in cancer, there is no doubt that miRNAs play a key role in the initiation and progression of cancer. Specific miRNAs have been demonstrated to regulate known oncogenes or tumor suppressor genes or act as so called onco-miRs or tumor suppressor-miRs by directly targeting other genes involved in cell differentiation, proliferation, invasion, apoptosis and angiogenesis in various cancers.

Because miR-30a-5p expression is up-regulated in glioma cell lines and glioma specimens (data not shown), miR-30a-5p may contribute to gliomagenesis.

Bioinformatics analyses with HuMiTar, a sequence-based method for prediction of human microRNA targets [9], have predicted that several miRNAs, including miR-30a-5p, are involved in the post-transcriptional regulation of SEPT7.

SEPT7 is a member of the septin family, which is a highly evolutionarily conserved subfamily of GTPases, consisting of at least 13 human septin genes that play important roles in cytokinesis, vesicle trafficking, polarity determination, microtubule and actin dynamics and can form membrane diffusion barriers. Septins have also recently been shown to be involved in oncogenesis [10]. SEPT7 has an open reading frame of 1254 nucleotides encoding 418 amino acids, including a GTP-binding motif, located on chromosome 7p14.4-14.1 [11]. Our previous study on the expression of SEPT7 in glioma cell lines and samples by mircroarray, RT-PCR, Western blotting and immunohistochemical staining demonstrated that SEPT7 gene expression was negatively correlated with the ascending order of glioma grades [12]–[14]. Moreover, we observed that enforced overexpression of SEPT7 inhibited cell proliferation, arrested the cell cycle at G0/G1 phase, and induced cell apoptosis *in vitro* and *in vivo* [14]. In addition, we showed that SEPT7 overexpression suppressed the invasion and migration ability of human gliomas, reversed the imbalanced state of MMPs/TIMPs, downregulated the expression of integrin alpha(v)beta(3) and altered the structure of tubulin-alpha [15]. These data strongly supported that SEPT7 is an important molecule in gliomagenesis, and should be considered as a tumor suppressor.

In the current study, we demonstrate that miR-30a-5p regulates the tumor-suppressive gene-SEPT7 as target gene, and suppression of miR-30a-5p directly lead to up-regulation of SEPT7. The effect of miR-30a-5p mimics promoting cell proliferation and inhibition of apoptosis can be reversed by enforced overexpression of SEPT7 in glioma cell lines.

## Materials and Methods

### Cell Culture

Human glioblastoma cell lines SNB19 and LN229 were purchased from the Institute of Biochemistry and Cell Biology, Chinese Academy of Science. All cells were cultured in Dulbecco’s Modified Eagle’s medium (DMEM) (Gibco, USA) supplemented with 10% fetal bovine serum (Invitrogen, USA) at 37°C in 5% CO2, and subcultured every 2–3 days.

### Oligonucleotides and Cell Transfection

The miR-30a-5p antisense oligonucleotides, mimics as well as scramble miRNA were obtained from Gene Pharma Co, Ltd (Shanghai, China), Their sequences were listed as follows: antisense-miR-30a-5p(30a-5p AS):5′-CUUCCAGUCGAGGAUGUUUACA-3′,miR-30a-5p mimics(30a-5p m):5′-UGUAAACAUCCUCGACUGGAAG-3′ and scramble miRNA(scr ODN) : 5′-CAGUACUUUUGUGUAGUACAA-3′. Oligonucleotides (20 pmol/µL) were transfected into glioblastoma cells at 70% confluence using Lipofectamine 2000 according to the manufacturer’s instruction (Invitrogen, USA). SEPT7 recombinant adenovirus (Ad-S7) was preserved by our laboratory.

### qRT-PCR Analysis of miRNA Expression

Total RNA from glioblastoma cells was isolated using Trizol reagent (Invitrogen, USA) for mRNA and miRNA analysis. For analysis of miRNA expression, real-time RT-PCR analysis was carried out. Amplification reaction was performed with MJ-real-time PCR (Bio-Rad, Hercules, CA, USA) using Hairpin-itTM miRNAs qPCR Quantitation Kit according to the manual. Relative gene expression was calculated using the 2^ΔΔCT^ method [16] and analyzed initially using Opticon Monitor Analysis Software V2.02 software (MJ Research, Waltham, MA, USA), normalized to the expression of U6. All qRT-PCRs assays were performed in triplicates, and the data are presented as means ± standard errors of the means (SEM).

### In situ Hybridization

Using antisense locked nucleic acid (LNA)-modified oligonucleotides probe, in situ hybridization was performed with In situ hybridization kit (Boster Biol Sci Co, Wuhan, China). The sequence of LNA-miR-30a-5p was 5′-CTTCCAGTCGAGGATGTTTACA-3′, scr ODN sequence was GTGTAACACGTCTATACGCCCA, and U6 ODN sequence was CACGAATTTGCGTGTCATCCTT. At 48 h after transfection, glioma cells were fixed with freshly prepared 4% paraformaldehyde (containing 0.1% DEPC). In situ hybridization detection of miR-30a-5p in GBM cells was conducted according to the protocol of the manufacturer. The fixed glioma cells were incubated with 20 µL LNA-miR-hybridization solution at 42°C for 16 h, and Cy3-avidin was used to label miR-30a-5p at a concentration of 0.5 mg/mL. Nuclei were counterstained with DAPI karyotyping kit (Genmed, Boston, MA, USA) and visualized using FluoView Confocal Laser Scanning Microscopes-FV1000 (Olympus, Tokyo, Japan) and analyzed using IPP5.1 (Olympus).

### Plasmid Constructs and Luciferase Reporter Assay

The human 3′-UTR of the SEPT7 gene which contains the putative binding site for miR-30a-5p, was amplified by PCR using the following primers carrying XbaI sequence: forward: 5′-CCTCTAGATTTTTTATT AAA-3′ and reverse: 5′-CCTCTAGAATTGTAATTATC-3′. The product was digested using XbaI enzyme and cloned into the XbaI treated PGL3-control vector (Promega, USA), then the 3′-UTR of the SEPT7 just located at the region immediately downstream of the luciferase gene in the reporter gene vector. The ligated product was transduced into E. coli JM109 and colony PCRs were used to screen for the clones harboring the forward-oriented insert, The desired construct was subsequently sequenced to obtain the vector PGL3-SEPT7-3′-UTR(PGL3-S7).

For the luciferase reporter assay, the human glioblastoma cell lines SNB19, LN229 were cultured in 96-well plates. They were transfected with 0.2 µg each of the PGL3 or PGL3-S7 plasmids and 5 pmol of the 30a-5p AS using Lipofectamine 2000. At 48 h after transfection, luciferase activity were measured using the Luciferase Assay System (Promega, USA).

### Cell Proliferation Assay

SNB19 and LN229 cells were seeded into 96-well plates at 4000 cells per well. After transfection as described previously, on each day of consecutive 7 days, 20µL MTT (5 mg/mL) was added to each well and the cells were incubated at 37°C for additional 4 h. and the supernatant was discarded. The reaction was then terminated by lysing the cells with 200µl of DMSO. Optical density was measured at wavelength of 570 nm and expressed as percentage of control. The data are presented as the mean ± SEM, which were derived from triplicate samples of at least three independent experiments.

### Flow Cytometric Analysis of Cell Cycle Kinetics

For analysis of cell cycle kinetics by flow cytometry, transfected and control cells in the log phase of growth were harvested, washed with PBS, fixed with 90% ethanol overnight at 4°C, and then incubated with RNase at 37°C for 30 min. Nuclei of cells were stained with propidium iodide for additional 30 min. A total of 10,000 nuclei were examined in a FACS Calibur flow cytometer (Becton-Dickinson, USA) and DNA histograms were analyzed by Modifit software.

### Measurement of Apoptosis by Annexin V staining

Parental and transfected cells were harvested at 48 h post-transfection. The apoptosis was analyzed by using AnnexinV FITC Apoptosis Detection Kit (BD Biosciences, USA) according to the manufacturer’s instruction. Annexin V-FITC and propidium iodide double staining cells detected by FACSCalibur were evaluated as the apoptotic cells [17]. The data obtained were analyzed with CellQuest software.

### Cell Invasion Detected with Transwell Assay

For analyzing the invasive activity of GBM cells, the upper surface of the transwell filters was coated with matrigel. Cells in the logarithmic growth phase were harvested. Cells(1×10^5^) in 200 µL of serum-free DMEM were added into the upper chamber. A total of 600 µL of conditioned medium derived from tumor cell culture was used as a source of chemoattractant and placed in the lower chamber. After 24-hour incubation at 37°C, the filters were gently taken out, the medium was removed from the upper chamber. The noninvaded cells on the upper surface of the inserted filter were scraped off with a cotton swab. The cells that had migrated into the lower surface of the inserted filter were fixed with methanol. The number of cells invading through the matrigel was counted using three randomLy selected visual fields under inverted microscope.

### Western Blot Analysis

At 48 h after transfection with oligonucleotides, total proteins from the parental and transfected cells were extracted and the protein concentration was determined by Lowry method. A total of 40 µg protein lysates from each sample was subjected to SDS-PAGE on 10%SDS-polyacrylamide gel. Separated proteins were transferred to a PVDF membrane (Millipore, USA). The membrane was incubated with primary antibodies against SEPT7, PCNA, Cyclin D1, Bcl2 and MMP9 (1∶1000 dilution, Santa Cruz, USA) followed by incubation with HRP-conjugated secondary antibodies(1∶1000 dilution, Zymed, USA). The specific protein was detected using a SuperSignal protein detection kit (Pierce, USA). After washing with stripping buffer, the membrane was reprobed with antibody against β-actin (1∶1000 dilution, Santa Cruz, USA). The band density of specific proteins was quantified after normalization with the density of β-actin.

### Immunofluorescence Staining

For immunofluorescence staining, control and transfected cells were seeded on coverslips and fixed with 4% paraformaldehyde (Sigma), treated with 3% H_2_O_2_ for 10 min and incubated with the primary antibodies described above overnight at 4°C. FITC- or TRITC-labeled secondary antibody (1∶200 dilutions) was added for 2 h at 37°C. DAPI reagent was used to stain the cell nuclei and the cells was visualized using FV-1000 laser scanning confocal microscopes and analyzed using IPP5.1 (Olympus).

### Statistical Analysis

Data were expressed as means ± SEM. Statistics was determined by ANOVA and χ^2^ test using SPSS11.0 (Windows). Statistical significance was determined as P<0.05.

## Results

### 30a-5p AS Specifically Knocks Down miR-30a-5p Expression

To evaluate the significance of miR-30a-5p overexpression in glioma cells, we used a loss-of-function antisense approach. miR-30a-5p antisense oligonucleotide was used to knock down miR-30a-5p expression in glioma cells. qRT-PCR results showed that the relative expression level of miR-30a-5p in 30a-5p AS treated SNB19 cells was 24.12±0.06% (P<0.05), and 19.02±0.04% in LN229 cells (P<0.05) compared with that in their control cells, respectively (Figure 1A). Furthermore, in situ hybridization demonstrated that the Cy3 red fluorescence signal in 30a-5p AS transfected SNB19 and LN229 cells was lower in contrast to the signal in control cells and cells transfected with scr ODN (Figure 1B). These data suggested that 30a-5p AS was able to inhibit specifically the endogenous miR-30a-5p expression in SNB19 and LN229 cells.

**Figure 1:** MiR-30a-5p expression was suppressed by 30a-5p AS in SNB19 and LN229 cells. MiR-30a-5p expression was knocked down in SNB19 and LN229 glioma cells compared with control by real time PCR (A) and In Situ Hybridization. (B).

### 30a-5p AS Suppresses Cell Proliferation

The proliferation of glioma cells *in vitro* was determined by MTT assay. As shown in Figure 2A1 and 2A2, 30a-5p AS treated SNB19 and LN229 cells showed a significant decrease in viability compared with the control and scr ODN transfected cells (*P*<0.05, from day 2 to 7). We found that the growth-inhibitory effect of 30a-5p AS reached maximum at 7th day, the end of observation period. The lowest survival rate was 50.88±6.28% for SNB19 cells, and 59.23±2.97% for LN229 cells.

**Figure 2:** 30a-5p AS suppressed glioma cell growth in SNB19 and LN229 cells. (A) The viability of glioma cells transfected with 30a-5p AS was decreased gradually during the 7-day observation period compared with control group and scramble groups determined by MTT assay in SNB19 cells and LN229 cells. (B) Flow cytometry data represented that S-phase fraction was much lowered and more cells were arrested in G0/G1 phase in the 30a-5p AS group compared with control and scramble groups. (C) Apoptotic Index (AI) of control and transfected SNB19 and LN229 cells was examined by Annexin V staining. As compared with the control and scramble group, the AI of the 30a-5p AS group cells was increased. (D) Invasive capability of parent and treated SNB19 and LN229 cells was examined by Transwell assay. Cell invasion was decreased in 30a-5p AS group compared with the control and scramble groups as assessed by the number of cells invading into the lower surface of the polycarbonic membrane via the matrigel.

### 30a-5p AS Arrests Cell Cycle in the G0/G1 Phase

To further analyze whether decreased viability effect of 30a-5p AS on SNB19 and LN229 was a result of cell-cycle arrest, the cell-cycle kinetics was analyzed using flow cytometry. Treatment with 30a-5p AS resulted in a decrease in the population of cells that were in S phase (Figure 2B1 and 2B2). A representative experiment was shown in SNB19 cells that S phase cell population accounted for 27.7±4.2% and 28.1±1.2% in control and scr ODN treatd groups, respectively, in contrast to 19.5±5.2% in 30a-5p AS treated cells. Similarly, the percentage of S phase cells decreased from 31.4±3.1% of control and 34.1±4.1% of scr ODN groups to 21.4±4.8% of 30a-5p AS group in LN229 cells. Compared with control and scramble ODN cells, the 30a-5p AS treated cells substantially and consistently increased the G0/G1 cell population from 50.9±3.4% of control group and 51.2±6.3% of scr ODN group to 61.1±3.2% in 30a-5p AS treated SNB19 cells. LN229 cells exposed to 30a-5p AS also arrested in the G0/G1 phase (60.2±5.5%) as compared to the control and scr ODN treated cells (49.1±3.1% and 48.2±3.2%, respectively), indicating that 30a-5p AS functions as a negative regulator of the cell cycle from G1-to-S transition.

### 30a-5p AS Induces Apoptosis

The effect of decreased miR-30a-5p on apoptosis was analyzed by conducting Annexin V and PI double staining. Untreated cells served as a negative control. Percentages of apoptotic cells are shown in the histogram (Figure 2C1 and 2C2). Compared with the apoptotic cells in control group (3.24±0.56% and 2.52±0.43%) and scr ODN treated group (3.87±0.21% and 2.38±0.78%) in SNB19 and LN229 cells, respectively, the downregulation of miR-30a-5p resulted in a significant (p<0.05) increase of apoptotic cells in SNB 19 and LN229 cells (14.94±2.15% and 12.76±1.78%, respectively), indicating an induction of apoptosis in SNB19 and LN229 cells by transfection of the 30a-5p AS.

### 30a-5p AS Inhibits Glioma Cell Invasion

The inhibitory effect of 30a-5p AS on glioma cells invasion was assessed by the transwell assay. Representative micrographs of transwell cell invasion are shown in Figure 2D1 and 2D2. The number of cells invading through the matrigel in the 30a-5p AS group (21.4±10.3) was significantly decreased from those of the Control group (87.2±8.7) and the scr ODN treated group (85.6±9.4) in SNB19 cells. In LN229 cells, invasive activity were also inhibited in the 30a-5p AS group (18.4±8.9) compared with that of the control group (93.5±10.5) and scr ODN treated group (95.7±5.8).

### 30a-5p AS Affects the Expression of Relevant Proteins Examined by Immunofluorescence Staining and Western Blot Analysis

When miR-30a-5p was knocked down, the expression of SEPT7 was upregulated while the expression of PCNA, Cyclin D1, Bcl2, MMP2 and MMP9 downregulated in SNB19 cells and in LN229 cells (Figure 3A, 3B), which coincided with the results determined by MTT, cell cycle kinetics, apoptosis and transwell assay.

**Figure 3:** The expression of SEPT7, PCNA, CyclinD1, Bcl2, MMP2, MMP9 in parent and 30a-5p AS treated SNB19 and LN229 cells detected by Immunofluorescence and Western blotting. SEPT7(49kDa) was up-regulated while expression of PCNA(36kDa), CyclinD1(37kDa), Bcl2(26kDa), MMP2(63kDa), MMP9(92kDa) significantly down-regulated when the miR-30a-5p expression was inhibited.

### SEPT7 is a Target of miR-30a-5p

To explore the mechanism by which miR-30a-5p regulates cell proliferation, invasion and apoptosis, miRNA targets prediction databases were searched, including miRanda, Targetscan and HuMiTar [9], and found 3′UTR of SEPT7 containing the highly conserved putative binding sites of miR-30a-5p (Figure 4A). To verify SEPT7 is one of the target genes of miR-30a-5p, we constructed the PGL3-S7 plasmid containing 3′UTR of SEPT7 with miR-30a-5p putative binding site and conducted a reporter gene assay. As shown in Figure 4B, reporter assay revealed that reduction of miR-30a-5p led to a remarkable increase of luciferase activity in PGL3-S7 combined with 30a-5p AS transfected cells(4.73±1.16 fold for SNB19, 5.14±0.87 fold for LN229), whereas no change of luciferase activity was found in PGL3-S7 with scr ODN transfected cells(0.95±0.32 fold for SNB19, 0.97±0.25 fold for LN229) and PGL3-S7 transfected cells(1.00±0.00 fold for SNB19 and LN229). Moreover, Western blot analysis showed that SEPT7 expression was up-regulated in glioma cells treated with 30a-5p AS compared to the cells treated with scr ODN or control cells, whereas no difference at the mRNA level of SEPT7 expression was observed among 30a-5p AS, control and scr ODN groups (Figure 4C). These evidences indicate that miR-30a-5p directly modulates SEPT7 expression at the translational level by binding to 3′UTR of SEPT7.

**Figure 4:** SEPT7 was a direct target gene of miR-30a-5p. (A) Schematic representation of the putative binding sites in SEPT7 mRNA 3′UTR for miR-30a-5p. (B) PGL3-S7-Luc vector was transfected into SNB19 and LN229 cells with 30a-5p AS transfection and luciferase activity was significantly increased. The ratio of normalized sensor to control luciferase activity was shown. * P<0.05 compared with control group. (C) SEPT7 protein and mRNA level was detected by Western blot assay and RT-PCR in SNB19 cells and LN229 cells transfected with 30a-5p AS, SEPT7 protein expression was upregulated while SEPT7 mRNA expression without change.β-actin protein and mRNA expression were regarded as endogenous normalizer.

### Downregulation of miR-30a-5p Results in Reduction of Glioma Cell Growth that is Partly Reversed by Tranfection with Ad-SEPT7

Having established that glioblastoma-derived cell lines displayed decreased proliferation and invasiveness *in vitro* when miR-30a-5p expression was decreased or SEPT7 was increased, we sought to further identify the role of miR-30a-5p and its target SEPT7 in gliomagenesis. We examined the proliferation, cell cycle progression, apoptosis and invasiveness of glioma cells after being treated with miR-30a-5p mimics (30a-5p m), SEPT7 recombinant adenovirus(Ad-S7) and 30a-5p m combined with transfection of Ad-S7(30a-5p+Ad-S7).

The expression of SEPT7 was downregulated in SNB19 and LN229 cells tranfected with 30a-5p m and upregulated when transfected with Ad-SEPT7 as detected by Western blotting, and SEPT7 expression was moderately increased in the cells transfected with 30a-5p m+Ad-SEPT7(Figure 5).

**Figure 5:** The expression of SEPT7, PCNA, CyclinD1, Bcl2, MMP2, MMP9 detected by Western blotting. SEPT7 is up-regulatd in group treated with Ad-SEPT7, down-regulated in 30a-5p m group and moderate expression in 30a-5p m+Ad-S7 group. The expression of PCNA, Cyclin D1, Bcl2, MMP2 and MMP9 was downregulated in Ad-SEPT7 group while up-regulated in 30a-5p m group, and the increased expression of relevant proteins was partly reversed in 30a-5p m+Ad-S7 group in SNB19 cells and LN229 cells.

The miR-30a-5p m cells proliferated at the highest level while Ad-S7 cells at the lowest and 30a-5p m+Ad-S7 cells grew at the intermediate level(Figure 6A). Similarly, As shown in Figure 6B and Table 1, compared to the cell cycle analysis of control cells, the S phase fraction of the SNB19 and LN229 cells treated with 30a-5p m was markedly increased while G0/G1 fraction decreased, in contrast to the cells transfected with Ad-S7 in which S phase fraction was significantly decreased while G0/G1 fraction increased. In the cells treated with 30a-5p m+Ad-S7 the decrease of S phase fraction or increase of G0/G1 fraction was moderate. The overexpression of SEPT7 led to a increased apoptotic index(15.48±2.34% and 17.34±3.94%) in SNB19 and LN229 cells respectively (Figure 6C). The 30a-5p m+Ad-S7 group showed a result (2.77±0.67 and 2.19±0.48) between the 30a-5p m (1.23±0.34% and 1.25±0.28%) and control group (3.03±0.75% and 2.67±0.53%). Transwell assay demonstrated that the SNB19 and LN229 cells transfected with 30a-5p m migrated through matrigel were increased, 124.7±16.3 and 135.6±17.8, respectively. These figures were higher than those in control groups. The migrating cells in control SNB19 and LN229 cells were 82.2±10.7 and 90.3±9.5, respectively. Enforced overexpression of SEPT7 obviously attenuated the cell invasion, migrating cells in Ad-SEPT7 group were 25.6±7.3 in SNB19 and 19.6±7.7 in LN229 cells, respectively, whereas the migrating cells in the 30a-5p m+Ad-S7 group were moderately increased, i.e. 100.5±12.5 in SNB19 cells and 107.4±12.6 in LN229 cells, respectively (Figure 6D). The expression of PCNA, Cyclin D1, Bcl2, MMP2 and MMP9 was downregulated in Ad-SEPT7 group while up-regulated in 30a-5p m group in SNB19 cells and in LN229 cells (Figure 5). The protein expression coincided with the results mentioned above in cell proliferation, invasion and apoptosis.

**Figure 6:** Upregulation of miR-30a-5p resulted in promotion of glioblastoma cell growth that was reversed partially by Ad-S7. (A) The figure showed that 30a-5p m increased the cell survival rate at a significantly higher rate in SNB19 cells and LN229 cells, (B) accelerated the glioma cells from G0/G1 to S phase in SNB19 cells and LN229 cells, (C) decreased the apoptotic cells in the 30a-5p m group, (D) promoted the cell invasive ability. And Ad-S7 inhibited cell proliferation(A), arrested the cell cycle in the G0/G1 phase(B), induced cell apoptosis(C) and suppressed the cell invasive ability(D). While the results of 30a-5p m+Ad-S7 group showed that 30a-5p m promoted the glioma cell growth that was partially reversed by overexpression of SEPT7.

**Table 1:** 30a-5p m promotes cell cycle progression.

	Group	G0/G1	S	G2/M
SNB19	Control	51.3±3.4	22.1±2.7	26.6±3.1
	30a-5p m	36.7±2.1	52.6±2.3	10.7±1.8
	Ad-S7	64.2±3.1	15.5±2.1	20.3±2.6
	30a-5p m+Ad-S7	45.8±4.1	25.3±6.2	28.9±2.5
LN229	Control	49.4±2.6	20.3±2.8	30.3±3.1
	30a-5p m	38.8±6.4	38.1±2.7	23.1±3.3
	Ad-S7	65.2±4.2	12.2±1.8	22.6±1.9
	30a-5p m+Ad-S7	43.8±6.5	26.4±5.2	29.8±2.8

Glioma cell lines transfected with 30a-5p m demonstrated increased cell viability and invasion, promotion of cell cycle and decreased apoptosis in vitro (Figure 6A, B, C, D), whereas transfected with Ad-SEPT7 showed the inhibition of cell proliferation, invasion, cell cycle progression, and induction of cell apoptosis, just the same as we observed previously [14]. Combined transfection with 30a-5p m and Ad-SEPT attenuate the effect of 30a-5p m. Taking together, all these results indicate that the effect of 30a-5p m on promoting cell growth, invasion and induction of apoptosis was able to be reverted by SEPT7 to a considerable degree. More importantly, this evidence identifiy that miR-30a-5p affects the cell biological behavior is partially through the negative regulation of SEPT7.

## Discussion

GBM is a highly invasive tumor of the central nervous system. Currently available combined therapies offer only limited benefits for patients with glioblastoma. It is imperative to develop novel therapeutic approaches by better understanding the molecular mechanism of gliomagenesis.

Recent studies indicate that various miRNAs play important roles in the initiation and progression of cancer. miRNAs may function as tumor suppressors by down-regulating the expression of tumor-promoting genes, or may have oncogenic role by inhibiting the expression of tumor suppressor genes. Regarding to the role of miR-30a-5p in cancers, there are so far only very limited data available. There has been reported that miR-30a-5p is aberrantly expressed in thyroid cancer [18], [19], gastric cancer [20], colon cancer [21], [22] and squamous cell carcinoma of human head and neck (HNSCC) and esophagus (ECC) [23]. Moreover, the expression of miR-30a-5p in these cancers are not inconsistent. For example, miR-30a-5p is upregulated in HNSCC and ESC while downregulated in colon cancer. Even in thyroid carcinoma its expression is different between papillary thyroid carcinoma (PTC) and anaplastic thyroid carcinoma(ATC). It is upregulated in PTC and dowregulated in ATC. The underlying mechanism of the different expression in various type of cancer is not yet clear. As to the expression of miR-30a-5p in glioma, that has not been reported before. Our previous study on microRNA expression profiles in glioma cell lines with microarray has demonstrated that miR-30a-5p is highly expressed, subsequently we confirmed this finding in seven glioma cell lines and forty three freshly resected glioma samples with different grades. According to bioinformatic analyses, SEPT7 is one of the predicted targets of miR-30a-5p. SEPT7 is reduced expression and plays a tumor suppressor role in gliomagenesis as we demonstrated before[12]–[14]. So in the present study, we are attempting to further identify SEPT7 is regulated by miR-30a-5p and miR-30a-5p may exert its oncogenic role through regulation of SEPT7.

The luciferase reporter assay validated that miR-30a-5p directly regulates SEPT7 expression by the presence of a binding site for miR-30a-5p in the 3′UTR of SEPT7. Moreover, Western Blot showed obvious upregulation of SEPT7 in the 30a-5p AS group compared to control and scr ODN groups, whereas no differences at the mRNA expression of SEPT7 were observed among 30a-5p AS, control and scr ODN groups. These results indicate the inverse correlation between the expression of SEPT7 and miR-30a-5p in glioma cells and miR-30a-5p negatively regulates SEPT7 expression at the translational level. Therefore, SEPT7 is a direct target gene of miR-30a-5p.

Our previous study has demonstrated that SEPT7 is downregulated in human gliomas. Forced overexpression of SEPT7 was able to inhibit cell proliferation and invasion, arrested cell cycle in the G0/G1 phase and induced apoptosis both in vitro and in vivo.

In this study, it has shown that when miR-30a-5p is knocked down with antisense oligonucleotide in SNB19 and LN229 cell lines, cell proliferation, invasion and cell cycle progression are inhibited, and apoptosis is induced. Meanwhile, SEPT7 expression is up-regulated. So that SEPT7 seems to be one of regulatory mechanism involved in the role of miR-30a-5p contributing to gliomagenesis.

Because miR-30a-5p can target multiple genes, we sought to explore whether SEPT7 is the major effector of miR-30a-5p for the change of biological behavior in glioma cells. Following transfection with miR-30a-5p mimics, we observed that glioblastoma-derived cell lines in which miR-30a-5p expression had been up-regulated, cell proliferation and invasion was enhanced compared to untreated control cell lines. More importantly, we found that the increased glioma cell growth can be reverted to a considerable degree by transfection of SEPT7. These results suggest that SEPT7 plays a major role in miR-30a-5p affecting biological behaviors of glioma cells.

Our results also showed that after inhibition of miR-30a-5p with 30a-5p AS, not only the expression level of SEPT7 was upregulated dramatically, but also the expression of proteins involved in cell proliferation, cell cycle progression, invasion and apoptosis, including PCNA, CyclinD1, Bcl2, MMP2, MMP-9 were decreased while BCL2 increased. On the contrary, When miR-30a-5p was up-regulated by transfection with miR-30a-5p mimics, PCNA, CyclinD1, Bcl2, MMP2, MMP-9 were increased while BCL2 decreased, and these results was also able to be partially reversed by transfection of Ad-SEPT7.

As miRNAs have a key role in the development of cancer, it is conceivable that miR-mimetics (for downregulated miRNAs) or anti-miRs (for upregulated miRNAs) could emerge as new class of molecular targeted therapeutic intervention [24]. On the basis of the 30a-5p AS-mediated upregulation of SEPT7, it is logical to predict that anti-miR-30a-5p could function as an potential effective, alternative therapeutic regimen against glioma. **In addition to SEPT7, there may be other targets of miR-30a-5p that may contribute to the gliomagenesis which should be further explored.**
